# Suitability Assessment of Surface Water Quality for Irrigation: A Case Study of Modjo River, Ethiopia

**DOI:** 10.1155/2023/1482229

**Published:** 2023-01-27

**Authors:** Andinet Kebede Tekile

**Affiliations:** Adama Science and Technology University, Adama 1888, Ethiopia

## Abstract

Water quality change due to industrial pollution is one of the major environmental concerns in developing countries. The majority of industries in Ethiopia release their wastewaters into the nearby water bodies with limited or without any forms of treatment. The main objective of this study was to assess the suitability of Modjo River for irrigation use based on the assessment of salinity, reduced water infiltration rate, specific ion toxicity, and miscellaneous chemicals as water quality-related problems in irrigated agriculture. Water samples were collected from six sampling stations along the river, and the relevant physicochemical parameters were determined in the laboratory by the standard procedures. Besides, the sodium adsorption ratio (SAR) and irrigation water quality index (IWQI) were determined to evaluate the suitability of the river water for irrigation. Cluster and principal component analyses of the data set were carried out. The results of this study showed that the river water in the vicinity of industries was saline and thus affects sensitive crops. The SAR value varied from 57.6 to 122.3. The concentration of chromium in the lower reaches of the river was also above the standard value of 0.1 mg/L. Among the miscellaneous chemicals, concentration of potassium, carbonate, and bicarbonate at all the sampling stations were above the standard values set by FAO for irrigation use. Based on the computed IWQI of 30.6, Modjo River is in the medium class of suitability for irrigation. Effluents from industrial establishments, namely, tannery, abattoir houses, and poultry farms and domestic waste dumping, were identified as the main sources of water pollution in the study area. Based on the findings of the study, Modjo River water is not suitable for irrigation use without some forms of physical and chemical treatment.

## 1. Introduction

Global water scarcity is caused not only by the physical inadequacy of the resource but also by the progressive deterioration of water quality in many countries, reducing the quantity of water that is safe to use [1]. Combinations of various natural factors and anthropogenic activities in rivers and their catchments are affecting water qualities. Industrialization and urbanization take a heavy toll on fragile water supplies, creating both new demands and risks of pollution [2]. Industries draw water from rivers for their use and in return release wastewater to rivers, which contains suspended and dissolved solids, oil and grease, heavy metals, fluorides, phosphates, ammonia, acids, etc. that badly affect the quality of rivers [3]. Pollution causes the water to become unsuitable for irrigation uses, and it is difficult and expensive to treat to the acceptable quality for use. On the other hand, urbanization affects the hydrologic regime of catchments, and it has a profound influence on the quality of storm water runoff. Consequently, it alters water quality in receiving waters. In general, streams in urbanized areas are likely to have higher levels of oxygen demand, nutrients, and suspended solids [4].

With poor quality water, soil and cropping problems develop, and in turn, these will reduce yields unless special management practices are adopted to maintain or restore maximum production capability under the given set of conditions. The suitability of water, from a quality standpoint, is determined by its potential to cause problems. Water quality-related problems in irrigated agriculture are salinity, reduced water infiltration rate, specific ion toxicity, and miscellaneous [5]. A salinity problem related to water quality occurs if total quantity of salts in the irrigation water is high enough that salts accumulate in the crop root zone to the extent affecting yields. On the other hand, a permeability problem related to water quality occurs when the rate of water infiltration into and through the soil is reduced by the effect of specific salts or lack of salts in the water to such an extent that the crop is not adequately supplied with water and thus yield is reduced. Carbonates and bicarbonates can also affect soil permeability and must be monitored. Furthermore, a toxicity problem occurs when certain constituents in the water are taken up by the crop and accumulated. This is usually related to one or more specific ions in the water. As a final point, various other problems, such as excessive nutrients, related to irrigation water quality should be specifically noted.

Environmental pollution derived from domestic and industrial activities is the main threat to the surface water qualities in Ethiopia [6]. The majority of industries in the country discharge their wastewaters into the nearby water bodies with limited or without any form of treatment [7]. In agreement with this, Yohannes and Elias [8] stated that 90% of the industries located in Addis Ababa discharge their waste without proper treatment. With the ever increasing demand on irrigation water supply, farmlands are frequently faced with utilization of poor quality irrigation water. In many parts of Ethiopia, industrial effluents, which are disposed into surface waters and nonfunctional treatment plants, are used as a source of irrigation [9]. However, the continued application of poor quality irrigation water can reduce the yield of farmlands, and it may have effect on the farmers, the consumers of the products, and the environment [10–12].

Due to government development polices and strategies, irrigated agriculture, industrial development, and urbanization are growing rapidly in the study area, especially during the last decade. Many industries are established in and around Modjo Town, especially along Modjo River. However, waste collection and treatment systems are not in proportion to the development plans that their effect on irrigated agriculture is expected. Modjo River, which is used as liquid waste disposal system by nearby tanneries and other industries, contains chemical pollutants with concentrations surpassing the permissible levels set by the National Environmental Quality Standards [6, 13]. The unlimited use of toxic chemicals in modern tanneries and disposal of their effluents into water bodies may have detrimental effects on human health and the aquatic environment [14]. Based on literature survey, Modjo River water quality suitability assessment for irrigation use has not been done so far; thus, this study was conducted to address this research gap.

To attain the objective, the physicochemical properties of water in the reach between Modjo Town and Koka Dam and pollutant sources affecting the water quality were investigated. The study results will be important to make available irrigation water quality information for the systematic monitoring programs, to make regulators and water users aware of the facts, and, thus, to assist them in making knowledge-based decision. The water quality suitability for use was judged on potential severity of problems that can be expected to develop during long-term use. FAO water quality standards, which are accepted in both developed and developing countries for irrigation use, have taken social, economic, and environmental factors into account [5]. Besides, water quality management tools, which are appropriate to the complexity of the situation and to the available data, enable understanding the problem simply.

## 2. Materials and Methods

### 2.1. Study Area

The research was undertaken on the upper part of the Awash River Basin of Ethiopia, particularly in Modjo watershed (Figure 1), which lies at upstream of Koka Dam and which has latitude and longitude range of 8° 16′ to 9° 18′ N and 37° 57′ to 39°17′ E, respectively, with total area of 1420 km^2^. Modjo River is a tributary to Awash River, and it flows through Modjo Town, which is located 75 km East of Addis Ababa. The town is the administrative center of Lome district, which is in the Eastern Shoa zone of Oromia regional state, and it is one of the industrial zones in the country.

Generally, highlands and lowlands characterize the topography of Modjo watershed. The highlands, with an elevation range of 1790–3060 m a.s.l., occupy the northern and western part of the study area whereas the lowlands, on the southern and eastern, have altitude range of 1550–1800 m a.s.l. The Northern part of the basin has a steep slope of more than 15%. Major rainy season of Modjo watershed is between June and mid-September with a short monsoon rain in March and April. Rainfall is unevenly distributed throughout the year, and it also shows strong altitudinal variations. The annual average rainfall is 1069 mm. Mean annual temperature is around 20°C. The lowest temperature occurs during the main rainy season; however, seasonal temperature variation is not pronounced.

Open bushy woodland being the dominant, dense wood lands, grass land, and open shrub are the prominent types of vegetation that are found in the study area. The main land use categories are cultivation of annual crops and livestock grazing and urban centers. Crop production has got a lion's share of the existing land use than livestock rearing. Nevertheless, it is an essential part of agricultural practices to back up the crop production. Cereal crops are entirely based on rainfall; besides, root crops and vegetables are produced along Modjo River using irrigation system.

### 2.2. Sampling Sites and Methods of Data Collection

For the water quality analysis, sampling sites were purposively selected along the course of the river based on accessibility, safety, and especially considering pollution sources [6]. Thus, the selected sampling sites were mainly located downstream of industries which release effluents into the river. Six sampling sites were selected from the upstream to the downstream, along the water course passing in Modjo town, namely at downstream of, a bridge from an industrial discharge, another bridge with no industry closely, Ethiopia Leather Factory PLC effluent release, old Modjo-Awassa highway bridge, farm field and at the end of Modjo River before it joins Koka Reservoir (Table 1).

Composite samples were taken from the river, considering spatial variations. Based on the standard method of sampling [15], two liter size plastic sampling bottle was rinsed with sample water, filled to the brim, airtight, and kept under cold conditions. All sample bottles were stored in an ice box and delivered in a day to laboratory. The samples were kept in the refrigerator until laboratory analyses were conducted. All the analyses in this study were done in triplicate. Water sample was collected from three points (left, right, and center) to accommodate the river cross-sectional variation, in addition to the longitudinal variation. From each sampling points, one-third of the sampling bottle of water was taken and mixed in the plastic bottle to form composite for laboratory test.

### 2.3. Sample Analytical Methods

To assess the suitability of the water for irrigation, the major physicochemical parameters associated with water quality problems were assessed. For salinity problem, electrical conductivity (EC) or total dissolved solids (TDS); for infiltration, calcium, sodium, magnesium, and sulphate as well as EC; for specific ion toxicity, sodium, chloride, boron, and chromium; and for miscellaneous effects, nutrients (nitrate-nitrogen, ammonium-nitrogen, orthophosphate, and potassium), bicarbonate, carbonate, and pH were determined.

The physicochemical sample water quality parameters analyses were carried out in accordance to the respective standard method [15]. Water pH was measured using a pH meter by just inserting the glass electrode, which was calibrated by standard buffer solutions of pH 4, 7, and 10. The temperature of the water sample was measured, and adjustment was made accordingly, since pH measurement is influenced by temperature. YSI professional series product family (USA), pro 1030 conductivity meter was used to determine EC and TDS. Calcium and magnesium were determined by complexometric titration method. Sodium and potassium were analyzed by flame photometer technique. The flame photometer was calibrated with standard solutions of sodium and potassium using NaCl and KCl salts before determination of Na and K, in water sample, respectively. Chloride was measured by argentometric titration with standardized silver nitrate solution, using potassium chromate solution in water. Boron was tested by photometer method by adding tablet available for this to water sample. Ammonia, nitrate, and orthophosphate were measured using photometer, for which reagents are provided in the form of two tablets for maximum convenience. Carbonate and bicarbonate were measured based on unique colorimetric methods. Sulphate was determined by nephelometric test, based on a single tablet reagent containing barium chloride in a slightly acidic formulation. Chromium was measured with palintest chromicol method, which provides a measure of the hexavalent chromium, and Cr (VI) present in the sample.

Irrigation water permeability problems are associated with sodicity. The tendency for sodium to increase its proportion on the cation exchange sites at the expense of other cations, primarily calcium and magnesium, was estimated by the sodium adsorption ratio, SAR [5]. SAR is calculated from the Na^+^, Ca^++^, and Mg^++^ concentrations reported in meq/l from water analysis as follows:

(1) $$\begin{array}{c} SAR=\frac{{Na}^{+}}{\sqrt{{Ca}^{2+}+{\;Mg}^{2+}/2}}\text{.} \end{array}$$

The physicochemical properties were compared with standards set by FAO for irrigation uses, to check the suitability of the water.

On the other hand, to know the cumulative effect of the hazard groups, namely, salinity, permeability, the basic toxicity of the ions, the toxicity of the trace elements, and the different consequences on the quality of water used for irrigation, irrigation water quality index (IWQI) was determined. To compute the IWQI, a weight, ranging from 1 to 5, was assigned to each group, and then ratings were assigned for individual physicochemical parameters based on their effect category [5, 16, 17]. The IWQI was computed by documented mathematical methods given as follows [16, 17]:

(2) $$\begin{array}{c} IWQI=\overset{5}{\underset{i=1}{\sum }}G_{i}\text{,} \end{array}$$

where *i* is the hazard group, and *G* is contribution of each hazard groups.

The salinity hazard (*G*_*1*_) is the first category expressed by EC as follows:

(3) $$\begin{array}{c} G_{1}=w_{1}r_{1}\text{,} \end{array}$$

where w_1_ is the group weight, and *r* is the parameter ranking.

The second hazard group is the risk of permeability (*G*_2_), which is expressed by the combined relationship between EC and SAR, which is given as follows:

(4) $$\begin{array}{c} G_{2}=w_{2}r_{2}\text{,} \end{array}$$

where *w*_2_ and *r*_2_ are the weight and rating of this group, respectively.

The third group is the toxicity of specific ion (*G*_3_), which includes SAR and the concentration of Cl and B ions in water. It is calculated according to a weighted average of these parameters as follows:

(5) $$\begin{array}{c} G_{3}=\frac{w_{3}}{3}\overset{3}{\underset{j=3}{\sum }}r_{j}\text{,} \end{array}$$

where *j* is the cumulative index, *w* is the group weight, and *r* is the ranking of each parameter.

A toxicity of trace elements represents the fourth group (*G*_4_), which is estimated as a weighted average for the individual trace elements, as follows:

(6) $$\begin{array}{c} G_{4}=\frac{w_{4}}{N}\overset{N}{\underset{k=1}{\sum }}r_{k}\text{,} \end{array}$$

where *k* is the cumulative index, *N* is the number of individual trace elements, *w* is the group weight, and *r* represents the ranking of each individual parameter. However, the only analyzed trace element in this study is chromium. The index computation is designed to allow incorporating only the measured elements without causing any error in the analysis due to the nonmeasured ones.

The final group is the miscellaneous effects to sensitive crops (*G*_5_), which is represented by the concentration of nitrate-nitrogen, alkalinity, and pH as a weighted average and described as follows:

(7) $$\begin{array}{c} G_{5}=\frac{w_{5}}{3}\overset{3}{\underset{m=1}{\sum }}r_{m}\text{,} \end{array}$$

where *m* is the cumulative index, *w* is the group weight, and *r* is the ranking of each parameter.

The suitability of the water for irrigation was then judged as low, medium, and high, corresponding to IWQI values of <22, 22–37, and >37, respectively [16, 17].

### 2.4. Statistical Analysis Methods

Mathematical, statistical, and data analysis were done by using Microsoft Office Excel 2010 and Statistical Package for Social Sciences (SPSS software version 26). Multivariate statistics is a useful way to evaluate spatial variation in river water quality and to identify possible anthropogenic sources of water quality patterns at monitoring sites in the river. Piper plot, cluster analysis (CA), and principal components analysis (PCA) were used for data analysis of this study.

Cluster analysis (CA) is commonly used for statistical data analysis in water quality assessment. CA is a multivariate statistical technique, which allows the assembling of parameters based on their similarity. CA classifies objects, so that each object is similar to the others in the cluster with respect to a predetermined selection criterion, such as sampling sites and the water quality parameters themselves. In this study, hierarchical agglomerative CA was performed on the normalized data set by means of the Ward's method of linkage, using squared Euclidean distances as a measure of similarity. CA reliably classifies surface water quality, and the results can be used as a guide for developing sampling strategies for the future [18]. Cluster analysis gives a visual summary of intrarelationship among parameters, which is helpful for better understanding of governing factors [19].

On the other hand, principal component analysis (PCA) can reduce dimensionality to make better sense of data by identifying the most influential variables in the data. It is a powerful technique for pattern recognition that attempts to explain the variance of a large set of interlinked variables and transform them into a smaller set of independent variables called principal components. In order to classify the variations of water quality, fifteen water quality parameters were used. PCA was executed using normalized variables to extract significant principal components (PCs), and these PCs were subjected to Varimax rotation generating factors to further reduce the contribution of variables with minor significance [18, 19]. In PCA, eigenvalues greater than unity were generally considered to be significant and to contain most of the variability of the original data set.

## 3. Results and Discussion

### 3.1. Salinity

Salinity (total dissolved salt content) of the river samples was evaluated in terms of EC (dS/m). EC values of the river water downstream of the industrial effluents release points were 4.15 dS/m and 7.65 dS/m at stations 1 and 3, respectively. The values are higher than the prescribed limit set by FAO, and the water is severe for irrigation purpose (Table 2). With higher EC, less amount of water will be available to plants, even though the soil may appear wet. This is because plant can transpire pure water as useable plant water, and this might decrease dramatically with an increase in EC. Therefore, irrigation water with high EC reduces yield potential. Highly saline water may also lead to concentrations of some elements which can be toxic to plants, such as boron, sodium, and chloride [20].

The EC values for water samples from the remaining four sampling sites showed slight to moderate salinity hazard (0.70–3.00 dS/m) for irrigation purposes [5]. The direct effect of EC which reflect the status of water pollution was replicated on the values of TDS. High TDS will decrease the productivity of the irrigation system and gradually may result in loss of the farm land due to salt-affected soil problem.

Further assessment of salinity of the river water was made based on salinity rating and suitability for specific types of crops (Table 3). Thus, based on the sensitivity or tolerance of crops to salinity, decision is required on the type of crops to be irrigated with the river water. As the water salinity rating is high or very high near the industrial discharges, only saline tolerant crops can be irrigated, unless otherwise the industrial effluent water is properly treated before its release to the river.

### 3.2. Infiltration

The sodium concentration in this study was from 14.7 to 28.2 meq/l (Table 4). Even though the values were relatively high downstream of industrial releases, all the water samples analyzed had Na^+^ concentration within allowable limit of FAO standard, for irrigation use. Just like sodium, both calcium and magnesium concentration values of the laboratory test for the river were within the allowable limits, thus suitable for irrigation purpose as per the standard. The maximum magnesium value of 1.6 meq/l was recorded at the sampling point in the farm field; this might be due to the effect of agricultural chemicals. Besides, the sulphate values for Modjo River during the study were between 1.3 and 3.5 meq/l, which are also below the acceptable limit for irrigation purpose. The maximum sulphate value observed at Modjo at Ethio-Tannery was possibly contributed by industrial discharge. Therefore, individually, the permeability related chemicals are safe. Generally, Modjo River water can be used without restriction for irrigation based on the individual results of the infiltration related chemicals.

Sodium or alkali hazard of water for irrigation is determined by relative concentration of cations in a water sample, which is expressed as SAR. SAR dictates the suitability of water for irrigation use. It gives a reliable evaluation of irrigation water quality with respect to sodium hazard, since it is more closely related to exchangeable sodium percentages in the soil than the simpler sodium percentage [20]. The SAR values of this study were either close to or above the value set by the standard. The main reason behind high concentration of SAR was the presence of relatively high concentration of Na ion to Ca and Mg ions in the water. High sodium concentration in irrigation water leads to soil crusting, poor seedling emergence, poor aeration, and substantial decrease in soil permeability. A high percentage of sodium on irrigation water may stunt the plant growth, deflocculating, and reduce the soil permeability which directly affects the irrigation productivity and potential irrigation commands. Thus, attention has to be paid to the water quality before applying for irrigation uses to avoid irreversible consequences. The results of Table 5 show that waters from the study area fall within category 1 and 2, which are suitable for irrigation on limited soil types with potential for the development of harmful levels of exchangeable sodium, if counteractions are not taken.

Combination of SAR and salinity could also be used to assess irrigation water quality with regard to permeability problem [21]. The SAR value of this study was between 10 and 23.8, whereas the EC was between 1 and 7.65 dS/m. Thus, from Table 6, only a site can be used without restriction, and for the remaining areas, the degree of restriction for irrigation is slight to moderate irrespective of their different agricultural practices. Generally, the quality of Modjo River is good for irrigation; however, given the high %Na of the waters, permeability could be impaired in the future if sodium was retained in the exchange complex.

### 3.3. Specific Ion for Toxicity

Specific ion toxicity affects sensitive crops. Crop yields are affected when chloride is above the maximum allowable limit for irrigation water, which is 106.5 mg/L according to FAO standard. The observed chloride values of all samples were below the maximum limit. However, the chloride contents downstream of industrial discharges sampling sites are relatively high. The higher concentration indicates pollution by industrial waste intrusion into the river [22]. Based on the overall chloride concentration (Table 7), the river water is suitable for irrigation purpose. To emphasis on values above FAO limit, they are shown in Italic in Table 7.

The other specific ion, boron, is needed in relatively small amounts; however, if it is present in amounts appreciably greater than needed, it becomes toxic. The concentration of boron in the river during the study ranged from 0.04 mg/l at Bridge Two to 3.10 mg/L at the site downstream of the highway bridge sampling point. Thus, the concentration of boron at Bridge One, which is affected by the industry effluent, was slightly higher than the acceptable limit set by FAO for irrigation purpose. The values of the remaining sites were within the limit set by the standard.

The values of chromium ranged from 0.02–0.15 mg/L. The chromium values of sites at Ethio-Tannery, Highway Bridge, and Terminal were greater than allowable standards of chromium hexavalent (0.1 mg/L) for irrigation use. The highest value in station at Ethio-Tannery was due to releasing of untreated tannery effluent into the river after tanning process [23]. Metal compounds are not biodegradable that the concentration is not reduced at stations further downstream.

### 3.4. Miscellaneous Chemicals

The minimum and maximum pH values of 8.57 at the Farm field station and 9.45 at Modjo at Bridge One, respectively, were recorded (Table 8). Four out of the six sites had pH within the limit of FAO standard [5]. The pH values were varied among the different locations as a result of dilution effect and pollutant sources. The bicarbonate varied from 430 to 1100 mg/L in the river; it reached high value of 1100 mg/L at the industry effluent. Discharge from industries and domestic wastes from the town were the main sources responsible for higher bicarbonate concentration. Out of six sampled water, only station 2 was within the standard. Thus, majority of the river water was not safe and suitable for irrigation purpose in relation to bicarbonate as per the standard set by FAO [5], in which the maximum allowable concentration was 610 mg/L. Again, entries of Table 8, which are in Italic, are to emphasis that they are above the FAO limit.

As per the FAO standard of irrigation water, the maximum limit of carbonate is 6 mg/L. The carbonate concentration during the study in the river was 210 mg/L (at Bridge Two) and 320 mg/L (at Highway Bridge). Both industrial discharge samples result had higher concentrations than the remaining samples carbonate concentrations. The effluent from factories is the major cause of the high carbonate concentration in the river.

Generally, potassium concentration in natural water is very low; however, pollution may increase the concentration to measurable extent. The K^+^ value of the water samples was between 36.7 and 76.3 mg/L. The maximum amount was found at Bridge One. All the analyzed water samples had values of potassium above allowable limit of FAO Standard for irrigation use [5]. Hence, it was not suitable for irrigation use in terms of potassium concentration.

The concentration of nitrite in the river was from 0.003 mg/L at Bridge One (industry effluent) and Modjo at Highway Bridge to 0.056 mg/L at Bridge Two sampling points. The nitrite concentration of the river during the study was within the permissible limit of 1.6 mg/L that the river water is suitable for irrigation purpose in relation to nitrite as per the standard. The concentration was below acceptable limit, even in the farm field. The concentration of ammonia in the river during the study ranged from 0.01 mg/L at the terminal to 0.69 mg/L at Bridge Two sampling points. The relative maximum ammonia value observed at Bridge Two sample site could be due to dumping of domestic wastes of Modjo town to the river. The laboratory test indicated that values of all sampling sites, including the farm field and industries effluent, were far below the acceptable limit set by FAO for irrigation purpose [5].

The phosphate concentration of the river during the study ranged from 0.11 mg/L at Bridge Two to 0.6 mg/L at Highway Bridge sampling points. Even though the phosphate value of the farm field sampling site was higher than the values from the remaining sites, it is within acceptable limit of FAO for irrigation use [5]. The relatively high phosphate value observed was 1.7 mg/L at Modjo at Bridge One, which was due to the industry effluent draining to the river. The concentration of phosphate at all sampling points during the study period was within the acceptable limit of FAO for irrigation uses [5]. As a result, regarding to phosphate, the river is safe for irrigation purposes.

### 3.5. Irrigation Water Quality Index

In the stated technique of IWQI determination, each of the parameters are assigned a weighing coefficient of 1 to 5 such that the most and the least important groups in irrigation water quality are given the highest (5) and lowest (1) points. Salinity hazard is the most important factor in irrigation water quality assessment that it is given the highest priority whereas the miscellaneous effects to sensitive crops are generally considered as the least significant factor [16]. The overall Modjo River water suitability for irrigation purpose is determined (Table 9) to assess the cumulative effect of the five hazard groups. The computed IWQI value is 30.06, and the corresponding suitability class for irrigation is thus medium.

To summarize the chemical concentrations, a piper plot is prepared. Grouping of water by Piper diagram was done to show gathering of data points to show samples with similar composition. The piper plot of Modjo River (Figure 2) showed that the concentration of Na ion is comparatively higher, and HCO_3_^−^ + CO_3_, Cl, and SO4 concentrations are low at all the sampling stations during the study.

### 3.6. Cluster Analysis and Principal Component Analysis

Cluster analysis (CA) was used to group the similar variables and to identify specific areas of contamination. The cluster analysis, using Ward's method (linkage between groups) with square Euclidian distance as a similarity measure, was amalgamated into dendrogram plot.  Figure 3 shows the output of the hierarchical agglomerative CA using fifteen data sets of water quality parameters. Thus, after performing the CA, the parameters are grouped into three clusters, which are cluster_1 (NO_2_, Mg and NH_3_), cluster_2 (Cl, EC, PO_4_ and B), and cluster_3 (CO_3_, HCO_3_, K, Na, SO_4_, pH, Ca, and Cr). Cluster _3 has got three separate subclusters itself, as shown in the dendrogram. The groupings show association among parameters which can be traced by the pollution sources, such as domestic, agricultural, and industrial releases.

Principal component analysis was used to identify significant water quality parameters. An eigenvalue greater than 1 considered as criterion for extraction of principal components. From the results of the factor analysis, the first four eigenvalues were found to be higher than 1, which explained over 88% of the total variance in the dataset. The different factors, total variance, cumulative variance, and loadings for the four components derived from the PCA are shown in Table 10. Factor loadings were classified as strong corresponding to absolute loading value of greater than 0.75 [19]. From the four PCs, the first component accounted for 48% of the total variance and has strong positive loading on EC, sodium, bicarbonate, carbonate, chloride, potassium, and phosphate, indicating variability in physico-chemical sources.

### 3.7. Potential Pollution Sources

The major pollutant sources are due to anthropogenic factors, mainly discharge of wastewater from domestic and factories to the river. There are large number of industries, governmental and private commercial and service rendering organizations which release their discharge and dump their solid waste into the river without any form of treatment. Major sources of wastewater effluents of Modjo River include Kolaba, Shoa, and Ethio-tanneries, Gelan, Derartu, and Ethio-Japan textile industries which discharge their raw effluent directly into the river. Modjo oil mill factory which drain its effluent to Mojo River and abattoir houses and poultry farms, which operate in the catchments of the river, also releases their effluents into Modjo River. Therefore, the major pollutant sources of water quality of Modjo River, downstream of Modjo town, are beverages, metal and tannery industries effluent, oil factory discharge, abattoir houses, and poultry farms effluent and domestic waste dumping. Especially during low flow period, due to low dilution capacity of the river, their effect is significant.

## 4. Conclusions

Physicochemical assessment of Modjo River water quality was conducted based on parameters relevant to indicate the suitability of the river water for irrigation uses. Six water samples, from which two samples are right after industrial effluents join the river and a sample in a farm field, were collected. Even though most of the physicochemical parameter values were within permissible limit for irrigation purpose, some major parameters such as carbonate, bicarbonate, chromium, and potassium were above the maximum limit at all the sampling points. Thus, attention should be given to the type of crops grown by using the river water for irrigation.

Most industries, service rendering and commercial organizations found in and around the town have aligned their waste disposal pipe to the river and release without any form of treatment. Even though these sectors are very important for the country's economy and livelihood of its citizens, the wastes which are discharged directly into the river seriously hurt the quality of the river. Based on the result, the water quality of Modjo River represents a severe threat to public health and agricultural use.

In order to improve the existing water quality problem, government and other concerned bodies should set and enact discharge realizing fee and enforcement law. Besides, the federal and regional government environmental protection authorities and Awash Basin Authority should make regular and proper monitoring, evaluation, and controlling of industries' treatment plant efficiency and their untreated wastewater discharge before reaching into river. Based on the current status of the river water quality, the concerned body should provide necessary awareness and training for the water users. Finally, it is recommended to conduct a detailed study with seasonal variation to investigate the extent of pollution fully.

## Figures and Tables

**Figure 1:** Location map of study area.

**Figure 2:** Piper plot of Modjo River water quality.

**Figure 3:** Dendogram of cluster analysis according to water quality parameters of Modjo River.

**Table 1:** The sampling sites.

Sampling station no	Stations	Station ID	Coordinate (*X*, *Y*)	Altitude
1	Bridge one	AW-AUSK-MODJO-01	511967, 949854	1742
2	Bridge two	AW-AUSK-MODJO-02	511937, 949846	1736
3	Ethio-tannery	AW-AUSK-MODJO-03	507106, 933508	1691
4	Highway bridge	AW-AUSK-MODJO-04	502817, 931651	1597
5	Farm field	AW-AUSK-MODJO-05	503398, 931609	1593
6	Terminal	AW-AUSK-MODJO-06	503492, 931489	1591

**Table 2:** Values of EC and TDS for water samples of the river.

Salinity parameter	Sampling stations						FAO limit [5]
	1	2	3	4	5	6	

EC (dS/m)	7.65	0.99	4.15	1.76	1.75	1.73	3.00
TDS (mg/L)	5130	664	2780	1182	1164	1157	2000

**Table 3:** Irrigation water salinity ratings based on electrical conductivity (Source: [20]).

EC (dS/m)	<0.65	0.65–1.3	1.3–2.9	2.9–5.2	5.2–8.1	>8.1

Water salinity rating	Very low	Low	Medium	High	Very high	Extreme
Plant suitability	Sensitive crops	Moderately sensitive crops	Moderately tolerant crops	Tolerant crops	Very tolerant crops	Generally too saline

**Table 4:** Infiltration-related parameters of the study area.

Infiltration parameter	Sampling stations						FAO limit [5]
	1	2	3	4	5	6	
Sodium (meq/l)	28.2	14.7	28.1	21.1	21.3	21.4	40.0
Calcium (meq/l)	4.3	3.0	2.8	5.4	4.1	5.0	20.0
Magnesium (meq/l)	0.0	0.8	0.0	0.7	1.6	0.4	5.0
Sulphate (meq/l)	2.0	1.3	3.5	2.8	2.5	2.4	20.0
SAR	19.2	10.7	23.8	12.1	12.6	13.0	15.0

**Table 5:** SAR values based on general irrigation water category (Source: [20]).

SAR	Category	Description of category	Precaution and management suggestions
0–10	1	Low Na water	Little danger
10–18	2	Medium Na water	Problems on fine texture soils and sodium sensitive plants, especially under low-leaching conditions. Soils should have good permeability
18–24	3	High Na water	Problems on most soils. Good salt tolerant plants are required along with special management such as the use of gypsum
>24	4	Very high Na water	Unsatisfactory except with high salinity (>2.0 dS/m), high calcium levels, and the use of gypsum

**Table 6:** Guidelines for interpretation of potential effect of irrigation water quality by using EC_w_ and SAR together (Source: [5]).

			Degree of restriction on use		
			None	Slight to moderate	Severe
SAR 0–3	And	EC_W_	>0.7	0.7–0.2	<0.2
SAR 3–6		EC_W_	>1.2	1.2–0.3	<0.3
SAR 6–12		EC_W_	>1.9	1.9–0.5	<0.5
SAR 12–20		EC_W_	>2.9	2.9–1.3	<1.3
SAR 20–40		EC_W_	>5.0	5.0–2.9	<2.9

**Table 7:** Concentration of specific ion for toxicity in the study area.

Specific ion for toxicity	Sampling stations						FAO
	1	2	3	4	5	6	
Chloride (mg/L)	58.8	5.0	32.6	9.3	9.1	8.5	106.5
Boron (mg/L)	*3.10*	0.04	0.90	1.15	2.40	1.05	3.00
Chromium (mg/L)	0.02	0.04	*0.15*	*0.13*	*0.11*	*0.13*	0.10

**Table 8:** The concentration of miscellaneous chemicals in Modjo River

Miscellaneous chemical	Sampling station						FAO limit [5]
	1	2	3	4	5	6	
Nutrients							
NH_3_-N (mg/L)	0.24	0.69	0.1	0.42	0.01	0.01	5.00
NO_2_-N (mg/L)	0.003	0.056	0.023	0.003	0.046	0.020	1.600
PO_4_-P (mg/L)	1.70	0.11	0.64	0.39	0.70	0.60	2.00
K (mg/L)	*76.3*	*36.7*	*54.9*	*46.5*	*47.1*	*47.8*	20.0
CO_3_^2−^ (mg/L)	*540*	*210*	*350*	*320*	*320*	*310*	6
HCO_3_^−^ (mg/L)	*1100*	*430*	*700*	*640*	*640*	*630*	610
pH	*9.45*	*9.03*	8.89	8.74	8.57	8.72	6–9

**Table 9:** Classification of IWQI parameters for surface water samples.

Hazard group	Weight	Parameter	Range	Rating	Suitability	Sample (%)	*G*_*i*_
Salinity	5	EC (dS/cm)	<0.65	3	High	Nil	8.335
			0.65 ≤ EC ≤ 2.9	2	Medium	66.7	
			>2.9	1	Low	33.3	

Infiltration and permeability	4	EC (*µ*S/cm) with SAR	See Table 6	3	High	16.7	8.668
				2	Medium	83.3	
				1	Low	Nil	

Specific ion toxicity	3	SAR	<10	3	High	Nil	6.667
			10 ≤ SAR ≤18	2	Medium	66.7	
			>18	1	Low	33.3	
		Chloride (mg/L)	Cl^−^ < 140	3	High	100	
			140 ≤ Cl^−^ ≤ 350	2	Medium	Nil	
			Cl^−^ > 350	1	Low	Nil	
		Boron (mg/L)	*B* < 0.7	3	High	16.7	
			0.7 ≤ *B* ≤ 3.0	2	Medium	66.7	
			*B* > 3.0	1	Low	16.7	

Trace element toxicity	2	Chromium (mg/L)	Cr < 0.1	3	High	33.3	4.666
			0.1 ≤ Cr ≤ 1.0	2	Medium	66.7	
			Cr > 1.0	1	Low	Nil	

Miscellaneous effects	1	Nitrate nitrogen (mg/L)	NO_3_ < 5	3	High	100	1.722
			5 ≤ NO_3_ ≤ 30	2	Medium	Nil	
			NO_3_ > 30	1	Low	Nil	
		Bicarbonate (mg/L)	HCO_3_ < 90	3	High	Nil	
			90 ≤ HCO_3_ ≤ 500	2	Medium	16.7	
			HCO_3_ > 500	1	Low	83.3	
		pH	7.0 ≤ pH ≤ 8.0	3	High	Nil	
			6.5 ≤ pH < 7.0 and 8.0 < pH £ 8.5	2	Medium	Nil	
			pH < 6.5 or pH > 8.5	1	Low	100	

**Table 10:** Loadings of fifteen variables (*p* ≤ 0.001) on Varimax-rotated principal components.

Parameters	Components			
	1	2	3	4
EC	0.977	−0.145	−0.133	0.076
Sodium	0.864	0.404	−0.261	0.140
pH	0.695	−0.677	−0.211	−0.117
Bicarbonate	0.990	0.002	0.137	−0.005
Carbonate	0.990	0.027	0.134	0.000
Potassium	0.999	−0.016	0.023	0.036
Phosphate	0.961	−0.053	0.221	0.136
Nitrite	−0.692	−0.357	−0.005	0.623
Calcium	0.134	0.378	0.656	−0.636
Ammonia	−0.334	−0.757	−0.165	−0.399
Chromium	−0.320	0.917	−0.234	−0.049
Magnesium	−0.622	0.053	0.644	0.354
Boron	0.767	0.106	0.561	0.268
Sulphate	0.171	0.874	−0.382	0.065
Chloride	0.961	−0.159	−0.197	0.097
Eigen value	5.517	3.133	1.643	1.223
Total % variance	48.013	20.887	10.954	8.154
Cumulative % variance	48.013	68.9	79.854	88.008

## Data Availability

All data generated or analyzed during this study are included in this manuscript.
